The article "Efficacy of Acupuncture Combined with Rehabilitation Training for Intensive Care Unit-Acquired Muscle Weakness: A Protocol for a Randomized, Sham-Procedure-Controlled Clinical Trial" was published in 2021. Journal: Evid Based Complement Alternat Med.

# Efficacy of Acupuncture Combined with Rehabilitation Training for Intensive Care Unit-Acquired Muscle Weakness: A Protocol for a Randomized, Sham-Procedure-Controlled Clinical Trial

**DOI:** 10.1155/2021/3539651

**Published:** 2021-10-20

**Authors:** Yin Shou, Wei Jin, Lingling Zhuang, Chenxia Xue, Li Hu, Siwei Xu, Kaiyong Zhang, Huiru Jiang, Peng Liu, Bimeng Zhang

**Affiliations:** ^1^Department of Acupuncture-Moxibustion, Shanghai General Hospital, Shanghai Jiao Tong University School of Medicine, Shanghai, China; ^2^Department of Critical Care Medicine, Shanghai General Hospital, Shanghai Jiao Tong University School of Medicine, Shanghai, China; ^3^Department of Ultrasound Medicine, Shanghai General Hospital, Shanghai Jiao Tong University School of Medicine, Shanghai, China; ^4^Department of Rehabilitation Medicine, Shanghai General Hospital, Shanghai Jiao Tong University School of Medicine, Shanghai, China; ^5^Acumox and Tuina Research Section, College of Acumox and Tuina, Shanghai University of Traditional Chinese Medicine, Shanghai, China

## Abstract

To evaluate the efficacy of acupuncture combined with rehabilitation training in patients with intensive care unit (ICU)-acquired muscle weakness (ICUAW), a single-blinded, randomized, sham-controlled clinical trial is designed for execution. In total, 56 participants with ICUAW will be randomly assigned to the treatment and control groups with 28 participants in each group. The participants will be treated with acupunctures or sham procedures at LI15, LI11, ST36, GB34, and ST31, 5 times per week for a total of 20 sessions in 4 weeks while they will receive rehabilitation training. Patients will be followed up every month for 3 months after treatment. The primary outcomes include changes in quadriceps femoris muscle area, thickness, vastus intermediate muscle thickness, subcutaneous tissue thickness, and ultrasonic intensities of the rectus femoris. The secondary outcomes consist of the modified Barthel index score and the Medical Research Council total score. Participants' mechanical ventilation, the rate of detachment at the second week, the 28-day survival rate, and the occurrence of adverse reactions will be measured, and any side effects will be reported and recorded. Patient outcomes between the treatment and control groups will be compared and statistically tested. We anticipate that the therapeutic regimen of acupuncture combined with rehabilitation training would be more effective than the rehabilitation training alone for the treatment of the ICUAW. The findings of this study could help develop a better strategy for the treatment of the ICUAW disease and explore a clinical application of an acupuncture technique. Trial registration: Chinese Clinical Trial Register ChiCTR2000038779. Registered 30 September, 2020, https://www.chictr.org.cn/showproj.aspx?proj=62284.

## 1. Introduction

The intensive care unit (ICU)-acquired weakness (ICUAW) is a generalized muscle weakness complication developed during ICU admissions for which no other disease cause can be identified except for acute illness or its treatment. Approximately 40% of ICU patients with a history of at least 48 h of mechanical ventilation develop ICUAW. The disease affects peripheral and respiratory muscles, causing prolonged time of mechanical ventilation and hospital stay, increased hospital mortality, and chronic disability [1–5]. The mechanisms by which ICUAW develops are complex and involve functional and structural alterations in both the muscles and the nerves. Recovery from ICUAW typically takes several weeks or months, and muscle weakness in some patients can last for up to 2 years after discharge from the ICU. Because the pathogenesis of ICUAW is still unclear, there are no specific treatments. The current management of ICUAW includes an active treatment of the primary disease (e.g., sepsis), prevention of infection, control of high blood sugar, reduction of the duration of immobilization, and avoidance of other known risk factors, such as malnutrition, unnecessary application of corticosteroids and neuromuscular blockers, and early rehabilitation [6–8]. Thus, the development of easy-to-perform, more effective ICUAW-targeted interventions is needed for the prevention and treatment of ICUAW.

Acupuncture is a component of the traditional Chinese medicine that is practiced in China as well as abroad as a part of medical care for systemic disease treatment and is believed to work on the principle of the redistribution of “QI,” the life energy concept in Chinese. As per traditional Chinese medicine, diseases result from an imbalance or poor flow of QI. Acupuncture can cure the diseases based on the conduction of meridians and acupoints and following the application of certain operations to improve the flow of QI. In our previous studies, we found that ICU-acquired myasthenia is an acute polyneuromyopathy, and early rehabilitation exercise alone can only reduce physiological dysfunction. Based on our clinical experience on the treatment of various neuromyopathy diseases, we found that acupuncture therapy can improve patients' nerve function [9], restore their muscle atrophy [10] and muscle mass and strength [11], relieve their symptoms, shorten offline time and hospital stay, and improve the quality of patients' lives. In particular, it can significantly alleviate the obvious atrophy of lower limb muscle thickness and cross-sectional area of ICU patients with acquired muscle weakness [12, 13]. More recent studies have found that the combination of acupuncture and speech rehabilitation training improved the total response rate of stroke patients with dysarthria [14]. Based on these studies, we presume that acupuncture and moxibustion combined with rehabilitation training can synergize the effects and offer complementary advantages. The combined therapeutic strategy is superior to simple acupuncture and rehabilitation training alone for the prevention and treatment of patients with ICUAW. However, the efficacy of this therapeutic regimen has not been evaluated yet. To test this hypothesis, we designed a randomized controlled trial with a 3-month follow-up to evaluate whether acupuncture combined with rehabilitation training benefits the recovery of patients with ICUAW and planned to determine the temporal extent of this effect after last successful treatment.

## 2. Methods and Analysis

### 2.1. Design

A parallel-group, randomized, and single-blinded (outcome assessors) prospective clinical trial was designed according to the Consolidated Standards of Reporting Trials (CONSORT 2010) guidelines (Figure 1), Standards for Reporting Interventions in Controlled Trials of Acupuncture (STRICTA) [15, 16], and Standard Protocol Items—Recommendations for Interventional Trials (SPIRIT) statement (Figure 2) [17] and the SPIRIT checklist. Patients with ICUAW will be recruited from the Shanghai General Hospital, which is affiliated to the Shanghai Jiaotong University from October 2020 to September 2023. Participants will be screened based on the inclusion and exclusion criteria; briefed on the purpose, procedures, treatments, and possible risks of the trial; and informed of their rights to discontinue participation in the clinical study at any time point. Once participants will have signed the written consent forms, they will receive either 20 sessions of acupuncture plus rehabilitation training therapy or sham acupuncture plus rehabilitation training for 4 weeks. The study design flow chart and the schedule are presented in Figure 1 and Table 1, respectively. In this study, we will follow the methods of Shou et al. 2020 [18].

### 2.2. Modified Barthel Index (MBI) Score and Medical Research Council (MRC) Total Score

#### 2.2.1. Inclusion Criteria

Participants who would meet all of the following criteria will be enrolled in the study: (1) age >18 years, male and female patients diagnosed with ICUAW; (2) those who were previously admitted to ICU for more than 24 h; (3) acute physiology and chronic health disease classification system II (APACHEII) scores in the range of 8–20 points calculated based on the 12 admission physiologic variables and patient's age and chronic health, as described by Knaus et al. [19]; (4) patients with stable hemodynamics; (5) patients with mechanical ventilation, oxygen concentration [fraction of inspired oxygen (FiO_2_)] < 0.6, and positive end-expiratory pressure (PEEP) < 10 cmH_2_O; and (6) patients who would either themselves and/or their families voluntarily agree to participate in the study and provide signed informed consent.

#### 2.2.2. Exclusion Criteria

ICUAW patients who have or had suffered from any of the following conditions will be excluded from the study: (1) primary neurological and muscular diseases before admission, including brain and spinal cord injury, Guillain–Barre syndrome (GBS), and myasthenia gravis; (2) limb disability and limb instability fracture; (3) malignant tumors; (4) active bleeding; or (5) alcoholic patients who would not stop drinking during the trial.

#### 2.2.3. Elimination Criteria

Enrolled participants will be allowed to withdraw from the study after being subjected to the assigned treatment if they: (1) leave the clinical trial for any personal reasons, (2) experience severe adverse life events that require them to withdraw from the trial, (3) do not fully participate in the treatment or follow-ups, and (4) do not comply with the treatment or fail to provide the information required for evaluation.

#### 2.2.4. Ethics

The study was approved by the Ethics Committee of the Institute of Shanghai General Hospital, which is affiliated to the Shanghai Jiaotong University [(2020)98]. An informed consent form will be prepared and provided to the participants for obtaining their signatures (as stated earlier).

#### 2.2.5. Randomization and Blinding

Participants will be randomly assigned (in a 1 : 1 ratio) to either the treatment group or the control group based on blocked randomization using a randomization table. The table will contain, in a random order, all possible combinations of a small series of figures and assume that patients are randomly assigned to treatment or control groups with equal probability. The order of the interventions assigned to each block will be randomized. The process will be repeated for consecutive blocks until all participants would have been randomized. During the period when the participants will receive the first treatment, they will be given sequential treatment cards from independent researchers to ensure adequate concealment. All participants will be treated separately to prevent communication. Except for acupuncturists, all relevant parties will be blinded to the intervention groups. The implementation of treatments will be performed by two acupuncturists who will use patches prepared by operational assistants. The needles will be applied to every participant in the treatment and control groups. In addition, acupuncturists, operational assistants, and research nurses will be instructed to refrain from communicating with the participants regarding anything that would lead them to determine their group allocation. In addition, outcome evaluators and statistical analysts will be blinded and will not be involved in any part of the design and treatments during the trial.

#### 2.2.6. Acupuncture and Sham Therapy

All research assistants and licensed acupuncturists involved in the trial will receive a 2-day training prior to the onset of the study. Both treatments will consist of 20 sessions over 4 weeks, 5 times per week, and each for 30 min. We plan to treat the patients for 4 weeks because normally our patients would have stayed in ICU for 4 weeks. Briefly, patients will be asked to lie down in a supine position. After sterilization, the 0.25 × 40 mm acupuncture needles (Suzhou Tianxie Acupuncture Instruments Co., Ltd., Suzhou, China) will be inserted to the acupoints of the Jianyu (LI15), Quchi (LI11), Zusanli (ST36), Yanglingquan (GB34), and Biguan (ST31) using a neutral reinforcing and reduced manipulation technique. Each needle will be rotated until the patient experiences the “QI” feeling of soreness, heaviness, and the sensation of distension. The procedure for conducting will be standardized as shown in Table 2. Participants in the control group will receive sham needling at the same acupoints with nested blunt needles. All the procedures will remain the same as the one in the treatment group with the exception of the needles, which will be forced to pierce the fixed pad and reach the skin surface without penetrating the skin. All participants will receive regular rehabilitation training.

### 2.3. Health Education

The conscious participants will be explained about the condition and their current situations, encouraged to have a positive attitude, and will be provided timely feedback on the stability of their vital signs. We plan to divert their attention, arrange visits from their family members, solve their psychological barriers, and eliminate their fears.

### 2.4. Rehabilitation Training

#### 2.4.1. Strategy

Physicians will first assess the tolerance of the patients to rehabilitation treatment. They will repeatedly evaluate whether the patients' oxygen supplies meet the respective consumptions and the conditions of their neurological, respiratory, circulatory, and other systems to determine the exercise mode of rehabilitation. Generally, rehabilitation intervention will be conducted in accordance with the following conditions: (a) maintenance of response to stimulation, having measurable cognitive ability characteristics, understanding of certain commands such as those that instruct them to open/close their eyes, look at people, show their tongues, nod, frown, and others; (b) FiO_2_ < 60%, PEEP <10 cmH_2_O; and (c) lack of orthostatic hypotension symptoms or need to pump vasoactive drugs. All patients will be required to be free of deep-vein thrombosis before the onset of rehabilitation. Physiotherapists will also evaluate the joint range of motion, the muscle strength, tension and endurance, and the ability of activities of daily life prior to the development of a standardized rehabilitation plan.

Physical training will be gradually advanced as follows: passive joints on the bed ⟶ active joints on the bed ⟶ active activity at bedside ⟶ assistance to get out of the bed. These tasks will be conducted 5 days/week. Patients would move on to the next stage only after completing the previous stage of training. If the participant becomes intolerant during recovery or if there is a tendency to change, the training will be stopped immediately.

### 2.5. Passive and Active Motion of Limb Joints

For the participants in coma or continuous sedation and those with limb muscle strengths < Grade III, a passive motion of limb joints will be performed. If the patient muscle strength is zero, we will help them to passively move each joint in both directions 8 times/group, two groups/exercise, 2 times/day, without half normal ranges of motion. If the muscle strength is Grade I or II, we will move the patient's points 8 times/group in 2 directions, and 2 times/group, 2 times/day, based on a normal range of motion. Conscious patients will be encouraged to exercise according to the following regime: clenched fist and double upper limb lifting exercise, double lower limb flexing 90°, straight leg raising 30°, 2 legs of alternate exercise for 10 min, 3 times/day; every 2 h the patients will be asked to turn over to lie on their sides and then sit upright on the bed (e.g., one end of the bed will be elevated). Patients will also be instructed to maintain the seated position if they can for 20 min, 3 times/day; otherwise, we will raise the head of the bed gradually and let the patients maintain the half-sitting position for 20 min, 3 times/day.

### 2.6. Sitting Position on and Beside the Bed

Conscious participants with upper limb muscle strengths of >Grade III will be provided with a back support to sit by the bedside for 10 min the first time, followed by 20 min the second time (provided they can tolerate it the first time), 2 times/day. They will also be helped to sit at the bedside for 1 h during the first-time exercise 2 times/day, followed by a gradually increase of up to 2 h if the patient can tolerate it the first time. The seating angle will be adjusted according to the participants' muscle strength.

### 2.7. Lower Extremity Muscle Exercises

Pet-type conditions will be added to lower extremity muscle exercises, such as bedside bicycle exercises. If the body and lower limb muscle conditions of the participants allow them to stand at the bedside but restrict them to walk, instruments for upper arm support will be provided, and the participants will be helped to stand at the bedside. For the participants with severe neuromuscular atrophy and those who cannot stand without support, “standing bed” will be used to help them stand up for 30 min/time, 2 times/day. For patients with muscle strengths of ≥Grade IV, the physiotherapist, physician, and nurse will coordinate their efforts and assist them to walk in the ward, 2 times/day. The walking distance will be determined according to the participants' tolerance.

### 2.8. Concomitant Care and Intervention

Participants with severe symptoms in both groups will be treated by first-aid kit medications. The type of medicine, dosage, and usage will be recorded on diary cards for analyses. For those with more complicated chronic diseases who must continue to take their routine medication and receive the necessary therapies, the names of the diseases, medications, and therapies used will be recorded.

Our registered nurses will monitor all the patients in the ICU 24 h/day, 7 days/week, and our ICU physicians will examine the patients every 6 h. In case the acupuncture causes hemodynamic instabilities, such as arrhythmias, hypotension, and confusion, the ICU physicians will be called immediately to treat the patients. In most cases, hemodynamic instability would require some type of artificial, mechanical support to maintain the blood pressure and heart activity. For cases in which the participants are unable to receive additional intervention with acupuncture rehabilitation after an evaluation, the participants will be withdrawn immediately from the study and undergo an alternative rehabilitation program. Based on our clinical experience, it is unlikely that patients will have sudden disorders of consciousness or limb twisting; these symptoms are usually experienced by patients suffering from seizures. If such problems arise in Grade I or II sectors of rehabilitation training, the patients will be kept away from the unsafe area and will be allowed to lie on their backs by removing the pillows. Any secretions from the mouth will be removed by turning the patients' heads to one side. Furthermore, ICU doctors will be called to rescue the patients and obtain neurological consultation.

### 2.9. Discontinuation of the Intervention

The intervention will be terminated in cases with severe adverse events, when participants wish to withdraw from the trial, or when patients use unpermitted medication that would interfere with the recovery outcomes. Patients will have the option to ask the doctor about possible alternative therapies (e.g., nutritional support such as use of tricreatine *β*-hydroxyl-methylbutyrate, antioxidant therapy, and immunoglobulin therapy).

### 2.10. Outcome Measures

#### 2.10.1. Baseline Information

Demographic information will be collected using a custom-made, standardized survey form that includes center location, name, age, gender, address, telephone number, and employment. Medical information will be collected using a custom-made form that records clinical information, including diagnosis, medication history, and APACHEII rating forms.

### 2.11. Primary Outcome Measures

The average change in the quadriceps femoris muscle area, thickness, vastus intermediate muscle thickness, subcutaneous tissue thickness, and ultrasonic intensity of the rectus femoris will be measured in a blinded manner, and the scores obtained at the baseline and at the end of the 4-week treatment will be compared for each group.

### 2.12. Secondary Outcome Measures

The average change in quadriceps femoris muscle area, thickness, vastus intermediate muscle thickness, subcutaneous tissue thickness, and ultrasonic intensity of the rectus femoris will be measured, and the scores obtained at the baseline, 2 weeks, and 3 months after the last treatment will be compared. MBI and MRC scores will be evaluated at 2 weeks, 4 weeks, and 3 months after the last treatment. The participants' mechanical ventilation, rate of detachment at the second week, 28-day survival rate, and occurrence of adverse reactions will be evaluated, and any noticed side effects of the treatment will be recorded. All outcome readings will be scored on quantitative scales and presented as mean values and standard deviations.

### 2.13. Safety Assessment

Adverse events (AEs) are defined as events in which at least four participants suffer from the same symptom, including any undesirable experiences that may occur during the trial period. This may or may not be associated with the intervention. Participants will be instructed to report any AE to the research team at any time. All details of AE, including the time of occurrence, description of symptoms, duration of symptoms, severity, management measures, and causality to the intervention, will be recorded on case report forms (CRFs). The common AEs related to acupuncture, including local skin pain, itching, ulcers, leaving needles in participants, nausea during acupuncture, fainting during acupuncture, severe sharp pain, sharp pain lasting for more than 30 min, hematomas around the site of needling, bleeding, numbness, infection around the needle sites, sleeplessness after acupuncture, and dizziness after acupuncture, will be reported [20]. The causality between AEs and intervention will be assessed according to the World's Health Organization Uppsala Monitoring Center System for Standardized Case Causality Assessment [21]. In the event of AE occurrence, patients will be given an appropriate treatment until their conditions stabilize. Severe AEs will be reported to the safety monitoring board within 24 h.

### 2.14. Follow-Up

The health statuses of the participants after the 4-week treatment period will be followed up on a monthly basis via telephonic and message communications for 3 months based on the previous study for this disease [22]. The symptoms and medication compliance or changes in medication will be recorded. In the event that participants withdrew from the trial or deviated from the intervention protocols, the staff will record the reasons for their withdrawal and the details of their new medications as well as the latest outcome data including the symptoms and frequency of the attacks prior to their exclusion from the study.

### 2.15. Participant Timeline

An overview of the recruitment timeline, interventions, and all time points of participant evaluation is summarized in Figure 2.

### 2.16. Data Collection and Management

The study staff will be responsible for the collection of baseline characteristic data and medical results during the screening period. All participants' scores, observation times, AE records, and safety assessments will be consolidated in a single CRF. CRFs will be filled out immediately and accurately. Outcome evaluators will examine the outcomes at the baseline (before the treatment), 2 weeks (during the treatment), 4 weeks (end of treatment), and 3 months after last treatment (during the follow-up period). Data monitoring and management will be performed every 3 months by the Clinical Research Center of the Shanghai General Hospital affiliated to the Shanghai Jiaotong University. The clinical research monitors will monitor the medical practitioners to ensure that all processes are implemented correctly. A data monitoring committee (DMC) independent of the sponsor and with no conflicts of interest will be responsible for monitoring the progression of the trial and ensuring patient safety. Interim analyses and trial discontinuation plans will not been specified, but will be provided upon DMC's request. Two assistants will enter all the data in an electronic database based on double data entry. The statistical manager will be responsible for data organization, coding, range checks for data values, and data conversion for quality control. The database will be locked after cleaning all data. If any participant withdraws from the trial, detailed reasons will be collected, and the rate of withdrawal will be analyzed statistically.

### 2.17. Quality Control

All the staff involved in the study, including acupuncturists, rehabilitation therapists, ultrasound examination doctors, operational assistants, and nurses, will be obliged to receive advanced training on filling out CRFs, conducting blood tests, details of acupuncture and rehabilitation therapy, scales and ultrasound examinations, and follow-up visit skills. All the staff members will be asked to take exams after training to ensure strict adherence to the study protocol and consistency of the trial administration processing, including acupuncture, rehabilitation therapy, and evaluation methods. All the staff members will be provided with a written protocol and standard operation procedure documents. All acupuncturists have acquired acupuncture licenses from the Ministry of Health of People's Republic of China; they must have a clinical experience of >5 years. To improve the quality of study reporting and conduct, we will develop a standard operating procedure manual according to the principles of the Consolidated Standards of Reporting Trials Extension for Chinese Herbal Medicine Formulas [23]; it will be explained to all the investigators. Intervention details, such as acpuncture rationale, details of needling, treatment regimen, time selection, practitioner background and confidence, and adequacy of stimulation, will be extracted and evaluated according to STRICTA [24]. To ensure the authenticity of the data, a special research team from the Clinical Research Center of the Shanghai General Hospital, which is affiliated to the Shanghai Jiaotong University and independent of the investigators and sponsors, will externally monitor the study in the hospital on a monthly basis. An advisory board will monitor the trial and provide advice when necessary. To improve adherence to the intervention, free 4-week treatments and examinations will be provided. To ensure that treatment and follow-up run as scheduled, participants will be given monetary compensation at the end of the follow-up period.

### 2.18. Statistical Analysis

#### 2.18.1. Sample Size Calculation

The trial will test two groups in parallel. The sample size calculation will be performed using the software SAS (version 9.3, SAS Institute Inc., Cary, NC, USA). The mean change in the primary outcome before and after treatment will be used as the indicator of efficacy evaluation in the calculation of the sample size. The results of previous studies yielded a mean ultrasound measurement of muscle thickness change of 0.45 ± 0.1 [25] and a mean ultrasonic intensity of muscle change of 25 ± 3 [26] after the loss of muscle mass and function. To detect a significant difference with a power of 80%, an alpha value of 0.05, and an acceptable delta value of 0.2, a sample size comprising at least 23 participants in each group will be needed. We have added an additional five patients per group considering a possible 20% dropout.

#### 2.18.2. Software for Statistical Analyses

Statistical analysis will be performed using SPSS (version 26.0, SPSS Inc., Chicago, IL, USA) in the Clinical Evaluation Center of Shanghai General Hospital, which is affiliated to the Shanghai Jiaotong University.

### 2.19. Sample Distribution

The size and dropout rate of each data set will be described. Detailed reasons related to participants' withdrawal from the trial will be provided.

### 2.20. Baseline Information

Baseline-adjusted analyses will be conducted for center and severity variables, and the baseline value of the corresponding outcomes will be assessed. Descriptive statistics will be used to compare baseline measures with participant characteristics. If an imbalance occurs in the baseline characteristics between the two groups, the analysis of variance will be applied.

### 2.21. Efficacy Analysis

Efficacy data analyses will be conducted based on the intention-to-treat population. All participants will be initially included in one of the two groups and considered in the statistical analyses. Analysis of efficacy will be conducted for each protocol and include all the participants who would complete the entire research processing. Descriptive statistics will be used to report primary outcome indicators between the two groups. All the data will be statistically analyzed using SPSS. All measurements will be expressed as mean ± standard deviation. The *t*-test will be used for comparisons between two samples if the distributions are normal, and the F-test will be used for comparisons among multiple samples. The Kruskal–Wallis H-rank sum test was used if the distribution is not normal. The participants' sex and course of disease will be recorded, and the data will be tested using the *χ*^2^ test. The ultrasound data will be analyzed by a mixed-effect model. The Cox-regression analysis will be performed to identify outcome-related factors. *P* < 0.05 will be considered as statistically significant.

### 2.22. Safety Analysis

According to the definition of AEs, AEs will be recorded in conjunction with their severity level, causes, and explanations. Moreover, the number and the rate of AE will be described statistically. If AEs would be required to be compared between groups, the *χ*^2^ test or the Fisher's exact test will be used for statistical analyses.

### 2.23. Missing Data Analysis

All data used in the main statistical analyses will be collected by the fourth week of the treatment and end of the 3-month follow-up period. If any of the data are not obtained, the assumed missing data mechanism will be analyzed, and a multiple adjustment approach will be used. After the main analysis, a sensitivity analysis will be performed for the various data sets to enable an assessment of the impact of the missing data on the results. A fully specified statistical analysis plan will be written independently.

### 2.24. Publication and Dissemination

Following the completion of data analyses, Chinese and English language disseminations will be planned. Trial results will be disseminated via conferences or publications. No public access will be provided to the entire protocol, participant data sets, or statistical code. However, scientists will be able to gain access to the full protocol through the Ethics Committee of the Institute of Shanghai General Hospital upon request. This protocol was written following the SPIRIT checklist. The future report will follow the CONSORT guidelines [13], revised STRICTA [12], and the extension of CONSORT for reporting single-blinded randomized trials.

## 3. Discussion

ICUAW is a frequent complication of critical illness, with devastating short- and long-term consequences. Therefore, effective prevention and/or treatment of ICUAW are required. Currently, the prevention of ICUAW development seems, at least in part, possible. However, to date, there is no effective therapeutic strategy to treat the disease [27, 28]. Some studies have shown that early rehabilitation has a positive effect on ICUAW recovery, shortens ICU and hospital stays, decreases the duration of mechanical ventilation, improves long-term functional independence, and reduces mortality [29–31]. However, a systematic review could not support the fact that post-ICU physical rehabilitation was beneficial because of the lack of high-quality data and existence of heterogeneity [32]. Another randomized controlled trial including 120 patients with acute respiratory failure found that the length of ICU and hospital stays were longer in the intervention group compared with those in the control group [33]. The early rehabilitation during ICU stay was not associated with improvements in functional status, muscle strength, quality of life, or healthcare utilization outcomes, although it seemed to improve walking ability compared with usual standard care [34, 35]. Thus, additional studies are required to design new preventive and/or therapeutic strategies that can be tested in adequately powered, large-scaled, well-performed, randomized controlled trials. Therefore, we developed the protocol of a randomized controlled trial presented herein to assess the effectiveness and safety of acupuncture combined with rehabilitation training for the treatment of patients with ICUAW.

Acupuncture is a feasible, safe, and acceptable therapy in ICU settings for patients with diversity backgrounds [36]. The therapeutic advantage of using acupuncture as an adjuvant therapy lies in the fact that the combination benefits the respiration of ICU patients on ventilation machine and helps weaning from prolonged ventilation [37]. The application of transcutaneous electrical nerve stimulation on acupuncture points has been shown to decrease the level of pain and opioid consumption in intubated patients connected to mechanical ventilators [38]. In addition, combined therapy of acupuncture with herbal medicine has been found to reduce the incidence of delirium in patients with cardiovascular disease in ICUs [39]. Furthermore, it is known that acupuncture with oral administration of essential amino acids is more effective and the combination can increase muscle mass in a relatively shorter time than treatment with the essential amino acids alone [11]. Recent studies have demonstrated that acupuncture can counteract skeletal muscle atrophy by increasing IGF-1 levels and by stimulating muscle regeneration [40]. In this report, we designed a single-blinded, randomized, sham-procedure-controlled, clinical trial with a 3-month follow-up for the assessment of the efficacy of acupuncture combined with rehabilitation training in patients with ICUAW. Successful completion of the proposed clinical trial will provide strong evidence that the therapeutic regimen of acupuncture combined with rehabilitation training is more effective than the rehabilitation training alone for the treatment of the ICUAW. The findings of this study could help to develop a better strategy for the treatment of the ICUAW disease and expand the application of acupuncture technique in clinical settings.

In this study, we proposed the use of muscular ultrasonography to evaluate the muscle strength by visualizing the muscle's cross-sectional area, layer thickness, and echo intensity based on the grayscale and penetration angle [41]. This is because the ultrasonic measurement of muscle thickness can be used to assess the presence of sarcopenia, and the echo intensity can be associated with muscle strength and correlated with the risk of frailty in elderly outpatients [25, 26]. We believe that muscle ultrasound can reliably detect the pathological changes of ICUAW [41]. Our study will address whether this treatment will affect the quadriceps femoris muscle area, thickness, vastus intermediate muscle thickness, subcutaneous tissue thickness, ultrasonic intensity of the rectus femoris, and MBI and MRC total scores in the long term after the last treatment.

## Figures and Tables

**Figure 1:** Flow chart of the study design.

**Figure 2:** Total study period and evaluation time points.

**Table 1:** Study design schedule.

Period	Baseline	Treatment (W1–W4)		Follow-up (W12)
Time	W0	W2	W4	W12
Eligibility	X			
Demography and medical history	X			
Physical examination	X			
Informed consent	X			
Quadriceps femoris muscle area	X	X	X	X
Quadriceps femoris muscle thickness	X	X	X	X
Vastus intermediate muscle thickness	X	X	X	X
Subcutaneous tissue thickness	X	X	X	X
Ultrasonic intensity of the rectus femoris	X	X	X	X
MBI	X	X	X	X
MRC	X	X	X	X
Adverse event			X	X
Compliance		X	X	

“X” indicates Yes. MBI: Modified Barthel Index; MRC: Medical Research Council.

**Table 2:** Acupoints and needle procedure.

Acupoints	Angle and direction	Depth (mm)
Jianyu (LI15)	Straightly	8
Quchi (LI11)	Straightly	8
Zusanli (ST36)	Straightly	13
Yanglingquan (GB34)	Straightly	13
Biguan (ST31)	Straightly	13

## Data Availability

The data used to support the findings of this study will be available from the corresponding author upon request.
